The article "MicroRNA-143-3p/TBX3 Axis Represses Malignant Cell Behaviors in Bladder Cancer" was retracted in 2023. Reasons: signs of a paper mill; suspected computer-generated content; unreliable results or conclusions; lack of ethics approval or compliance.

# MicroRNA-143-3p/TBX3 Axis Represses Malignant Cell Behaviors in Bladder Cancer

**DOI:** 10.1155/2022/2880087

**Published:** 2022-01-27

**Authors:** Lifu Huang, Xianjun Zhang, Feiping Li, Xiaohong Wang

**Affiliations:** ^1^Department of Urology, Taizhou Hospital of Zhejiang Province Affiliated to Wenzhou Medical University, Linhai, Zhejiang Province, China 318050; ^2^Enze Hospital, Taizhou Enze Medical Center (Group), Taizhou, Zhejiang Province, China 318050; ^3^Obstetrical Department, Taizhou Hospital of Zhejiang Province Affiliated to Wenzhou Medical University, Linhai, Zhejiang Province, China 318050

## Abstract

**Objective:**

To offer new insight for bladder cancer therapy through researching the microRNA-143-3p/TBX3 axis.

**Methods:**

Differentially expressed microRNAs in bladder cancer were provided by databases to find microRNA that may regulate TBX3. qRT-PCR was utilized to test levels of TBX3 mRNA and microRNA-143-3p. Their binding was verified with a dual-luciferase method. Malignant cell behaviors were examined by cell functional experiments. Levels of TBX3 protein and proteins pertinent to epithelial-mesenchymal transition (EMT) were tested by western blot.

**Results:**

TBX3 was highly expressed in bladder cancer cells. MicroRNA-143-3p presented the most conspicuously negative correlation with TBX3, and they had binding sites. Cell functional experiments proved that TBX3 facilitated bladder cancer cell functions and EMT. MicroRNA-143-3p was demonstrated to downregulate TBX3 expression. Rescue assay further illuminated that microRNA-143-3p repressed bladder cancer cell functions and EMT through downregulating TBX3 expression.

**Conclusion:**

These data all indicated that TBX3 was modulated by microRNA-143-3p and acted as a cancer promoter gene in bladder cancer progression via affecting tumor proliferation, migration, invasion, and EMT. Therefore, a microRNA-143-3p/TBX3 network might be an underlying target for bladder cancer.

## 1. Introduction

Bladder cancer is a prevalent malignancy in the urinary system [1]. Nonmuscle infiltrating bladder cancer comprises most of all bladder cancer cases (70%-80%) and shows a favorable prognosis [2]. Nonetheless, muscle infiltrating bladder cancer shows a terrible therapeutic effect, and the recurrence rate is high [3]. Generally, bladder cancer patients' median survival is rather short (10-55 months). A patient's poor prognosis often results from distant metastasis and high recurrence [4, 5], while epithelial-mesenchymal transition (EMT) facilitates invasiveness and activity of bladder cancer cells [6, 7]. Hence, it is critical to define the functional mechanism in the early stage of metastasis, such as migration, invasion, and EMT.

The article "MicroRNA-143-3p/TBX3 Axis Represses Malignant Cell Behaviors in Bladder Cancer" was retracted in 2023. Reasons: signs of a paper mill; suspected computer-generated content; unreliable results or conclusions; lack of ethics approval or compliance.

T-box protein family consists of a group of evolved conservative transcription factors which modulate levels of genes [8]. They work as transcriptional inhibitors or activators to modulate EMT, tissue integrity, and cell differentiation [9–11]. Overexpressing T-box factors such as TBX3 and TBX2 might trigger cancers [12–16], and these two transcription factors are activated in melanoma [17, 18] and bladder cancer [19, 20] and are proved to be necessary for tumorigenesis and migration [20, 21]. Furthermore, previous studies suggested that TBX3 expression promotes tumor EMT and TBX3 upregulation directly inhibits adhesion molecule E-cadherin expression, thereby increasing the aggressiveness of melanoma [22]. E-cadherin is an important medium of cell-cell interaction, which is verified to be significant in EMT, and loss of E-cadherin is the most crucial marker for EMT occurrence [23]. TBX3 is proved to promote proliferation and invasion and repress apoptosis of rat bladder cancer cells [24]. Conspicuously expressed TBX3 functions as an underlying indicator for bladder cancer diagnosis and/or prognosis [19]. An intriguing investigation also supports this result by identifying TBX3/TBX2 as a favorable marker for primary pTaG1/2 bladder cancer [25]. All these data lay stress on the importance of TBX3 as a potential biomarker. Nonetheless, how TBX3 functioned in the malignant progression of bladder cancer has been hardly known.

TBX3 was predicted as a target of microRNA-143-3p through bioinformatics methods. Therefore, this investigation is concerned with microRNA-143-3p/TBX3 in bladder cancer and the effect of their abnormal expression on tumor biological functions. Our results may lay a foundation for finding potential molecular therapeutic targets of bladder cancer.

## 2. Materials and Methods

### 2.1. Cell Culture

Human bladder cancer cell lines T24 (BNCC311582), BIU-87 (BNCC100982), and immortalized human bladder epithelial cell line SV-HUC-1 (BNCC100273) were bought from Bena Culture Collection (BNCC) (China). Human bladder cancer cell line UMUC3 (ATCC® CRL-1749™) was from American Type Culture Collection (ATCC) (USA). T24 and BIU-87 cell lines were treated in RPMI-1640 medium plus 10% fetal bovine serum (FBS). UMUC3 cell line was placed in DMEM with 10% FBS. SV-HUC-1 was cultured in CM7-1 medium containing 90%F‐12K + 10%FBS. All cell lines were cultured in a temperature incubator with 5% CO_2_ at 37°C.

### 2.2. Construction of Vectors and Transfection of Cells

MicroRNA-143-3p mimic, mimic NC, si-TBX3, si-NC, oe-TBX3, and oe-NC were designed by Guangzhou RiboBio. Lipofectamine 2000 (Thermo Fisher Scientific, Inc.) was applied to transiently transfect synthesized sequences or plasmids into bladder cancer cells T24 or BIU-87. Cells were incubated in corresponding mediums with 5% CO_2_ at 37°C for use. Before transient transfection, all cells were cultured for at least 24 h and needed to be washed with phosphate-buffered saline (PBS) (pH 7.4).

The article "MicroRNA-143-3p/TBX3 Axis Represses Malignant Cell Behaviors in Bladder Cancer" was retracted in 2023. Reasons: signs of a paper mill; suspected computer-generated content; unreliable results or conclusions; lack of ethics approval or compliance.

### 2.3. qRT-PCR

Total RNA was isolated from cells using TRIzol kit (Invitrogen, Carlsbad, CA, USA). RNA concentration was determined by NanoDrop 2000 system (Thermo Fisher Scientific, Inc., Waltham, MA, USA). Following the kit instruction, miScript IIRT kit (Qiagen, USA) was used to reversely transcribe microRNAs into cDNA, and mRNAs were reversely transcribed into cDNA by using PrimeScript RT Master Mix (Takara Bio Inc., Dalian, P.R. China). miScript SYBR Green PCR Kit (Qiagen, Germany) was used to detect microRNA expression and SYBR® Premix Ex Taq™ II (Takara Bio Inc., Shiga, Japan) was applied to detect mRNA expression. qRT-PCR was undertaken on Applied Biosystems®7500 Real-Time PCR Systems (Thermo Fisher Scientific, Inc., Waltham, MA).  Table 1 provides the used primers that were all purchased from Sangon Biotech (Shanghai, China). U6 and *β*-actin were taken as the internal references of microRNA-143-3p and TBX3, respectively. The difference of relative expression between groups was compared by 2^-*ΔΔ*Ct^ value.

### 2.4. Western Blot Assay

Cells were lysed with radioimmunoprecipitation analysis buffer (Sigma-Aldrich) containing protease inhibitor. Total proteins were determined by bicinchoninic acid (BCA) method (Sigma-Aldrich). Proteins were separated through 10% sodium dodecyl sulfate-polyacrylamide gel electrophoresis and then transferred onto a polyvinylidene fluoride membrane (Sigma-Aldrich). After being blocked with 5% skim milk at room temperature for 1 h, the membrane was incubated with primary antibodies overnight. Primary antibodies were rabbit anti-TBX3 (1 : 1000, ab154828, Abcam, UK), rabbit anti-E-cadherin (1 : 10000, ab40772, Abcam, UK), rabbit anti-N-cadherin (1 : 5000, ab76011, Abcam, UK), rabbit anti-Vimentin (1 : 1000, ab92547, Abcam, UK), and rabbit anti-*β*-actin (1 : 1000, ab8227, Abcam, UK). After being washed with PBS with Tween 20 3 times (each time for 10 min), the membrane was reacted with secondary antibody goat anti-rabbit IgG H&L coupled with horseradish peroxidase (HRP) (ab205718, Abcam, UK) for 1 h at room temperature. Enhanced chemiluminescence (Solarbio, Beijing, China) was added for development. Analysis was taken using the gel imager (Gel Doc XR, Bio-rad, USA), and grey scale value was processed by ImageJ.

### 2.5. Cell Counting Kit- (CCK-) 8 and Colony Formation Assays

In CCK-8, 2 × 10^4^ transfected cancer cells were placed into 96-well plates with each well (100 *μ*l medium). At 0, 24, 48, 72, and 96 h, 10 *μ*l CCK-8 (Dojindo, Tokyo, Japan) was added for another 1 h of incubation. Absorbance was measured with a microplate reader at 450 nm.

The article "MicroRNA-143-3p/TBX3 Axis Represses Malignant Cell Behaviors in Bladder Cancer" was retracted in 2023. Reasons: signs of a paper mill; suspected computer-generated content; unreliable results or conclusions; lack of ethics approval or compliance.

In colony formation assay, transfected bladder cancer cells were inoculated into 6-well plates at each well (1 × 10^4^) cells. Next, cells of each well were cultured in 2 ml medium for a week. Afterward, cells were washed with PBS twice, treated with 4% paraformaldehyde and 0.1% crystal violet for 20 min. Aggregates ≥ 50 cells (diameter: 0.3 mm-1 mm) were defined as colonies.

### 2.6. Detection of Migration and Invasion

Cell migration and invasion were examined by using Transwell cell migration chamber and BioCoat Matrigel-coated Transwell cell invasion chamber (Corning, NY, USA). After 24 h of transfection, T24 or BIU-87 cells were suspended in 200 *μ*l serum-free medium. Cell suspension was added into the upper chamber, and the lower chamber was covered with 500 *μ*l RPMI-1640 containing 15% FBS. Thereafter, cells were incubated at 37°C for 24 h. Next, cells in the upper chamber were removed. Cells in the lower chamber were treated with 4% paraformaldehyde for fixation and 0.5% crystal violet for staining. Under 5 randomly selected fields of the microscope (100x), migrating and invading cells were, respectively, counted.

### 2.7. Dual-Luciferase Reporter Detection

To identify the binding between microRNA-143-3p and TBX3 3′-UTR, mutant (MUT) (by site mutation), and wild-type (WT) TBX3 3′-UTR were constructed. Next, sequences were inserted into psiCHECK luciferase reporter plasmids (Sangon Co., LTD, Shanghai, China). Next, bladder cancer cells (T24) were inoculated in 48-well plates and cultured at 37°C for 24 h. T24 cells were transfected with microRNA-143-3p mimic or mimic NC and WT/MUT-TBX3 plasmids. Ultimately, luciferase activity was measured through a luciferase determination kit (Promega, Fitchburg, WI, USA).

### 2.8. Statistical Analysis

Data were exhibited as the mean ± standard deviation (SD) and processed by using GraphPad Prism 6.0 software (GraphPad Inc., San Diego, CA, USA). The difference between two groups was analyzed by a *t*-test and among more than 2 groups was analyzed by variance analysis. All experiments were repeated 3 times independently. *p* < 0.05 was defined as statistically significant.

## 3. Results

### 3.1. TBX3 Is Conspicuously Highly Expressed in Bladder Cancer

Combining reference analysis, TBX3 overexpression is relevant to many cancers, such as liver cancer, pancreatic cancer, ovarian cancer, and head and neck squamous cell carcinoma [26]. However, little is reported about the mechanism by which TBX3 modulates bladder cancer, and therefore, we chose TBX3 for research. Basic TBX3 level in T24, BIU-87, UMUC3, and SV-HUC-1 was tested first. It was unveiled that TBX3 expression was higher in cancer cells than in normal cells at mRNA and protein levels (Figures 1(a) and 1(b)). Hence, we considered that TBX3 was remarkably upregulated in bladder cancer. T24 and BIU-87 cells with a remarkable difference in TBX3 expression were used for the following experiments.

The article "MicroRNA-143-3p/TBX3 Axis Represses Malignant Cell Behaviors in Bladder Cancer" was retracted in 2023. Reasons: signs of a paper mill; suspected computer-generated content; unreliable results or conclusions; lack of ethics approval or compliance.

### 3.2. TBX3 Facilitates Bladder Cancer Cell Proliferation, Migration, Invasion, and EMT

Since TBX3 was conspicuously highly expressed in bladder cancer cells, this part is aimed at verifying its effect on the biological function of bladder cancer cells. Cells with TBX3 low expression and TBX3 high expression were constructed by transient transfection of si-TBX3 (si-NC as control) into T24 cells and oe-TBX3 (oe-NC as control) into BIU-87 cells, respectively. qRT-PCR was applied to detect transfection efficiency (Figure 2(a)). CCK-8 and colony formation assays indicated that silenced TBX3 remarkably inhibited T24 cell proliferation, while overexpressed TBX3 facilitated BIU-87 cell proliferation (Figures 2(b) and 2(c)).

Subsequent analyses were conducted to determine whether TBX3 impacted cancer invasion and migration. Transwell assay suggested that declined TBX3 expression suppressed T24 cell migration and invasion, while overexpressed TBX3 increased BIU-87 cell migration and invasion (Figure 2(d)). Furthermore, EMT-related proteins in different transfection groups were measured by western blot. An increase in E-cadherin level while a reduction in levels of N-cadherin and Vimentin was observed in si-TBX3-transfected T24 cells, and TBX3-overexpressed BIU-87 cells showed the opposite situation (Figure 2(e)).

### 3.3. MicroRNA-143-3p Downregulates TBX3 Expression

To further determine how TBX3 affects the malignant progression of bladder cancer, we predicted its upstream microRNAs. The predicted microRNAs by bioinformatics databases were intersected with differentially expressed microRNAs (DEmicroRNAs) from TCGA to acquire 7 candidate microRNAs (Figure 3(a)). Afterward, correlation analysis was conducted on the 7 microRNAs and TBX3, and it was displayed that microRNA-143-3p had the most significantly negative correlation with TBX3 (Figure 3(b)). Meanwhile, it was predicted that they had binding sites (Figure 3(c)). A dual-luciferase method confirmed that microRNA-143-3p overexpression declined luciferase intensity of WT TBX3 3′-UTR reporter plasmids, suggestive of their direct binding (Figure 3(d)). Thereafter, qRT-PCR discovered markedly low microRNA-143-3p levels in cancer cells (Figure 3(e)). Moreover, we constructed microRNA-143-3p overexpressed T24 cells and NC T24 cells. TBX3 expression in two groups was compared. Results exhibited that TBX3 mRNA and protein level in microRNA-143-3p mimic transfected T24 cells were significantly downregulated (Figures 3(f) and 3(g)). Overall, microRNA-143-3p was less expressed in bladder cancer and had negatively regulatory relationship with TBX3.

The article "MicroRNA-143-3p/TBX3 Axis Represses Malignant Cell Behaviors in Bladder Cancer" was retracted in 2023. Reasons: signs of a paper mill; suspected computer-generated content; unreliable results or conclusions; lack of ethics approval or compliance.

### 3.4. MicroRNA-143-3p Constrains EMT and Cell Functions via TBX3 Mediation

In the above context, we testified that microRNA-143-3p could downregulate TBX3 expression. Thereafter, to further scrutinize the microRNA-143-3p/TBX3 axis, we arranged rescue assays. MicroRNA-143-3p mimic was utilized to recover TBX3 expression (Figure 4(a)). As revealed by CCK-8 and colony formation methods, overexpression of TBX3 alone markedly stimulated cancer cell proliferation and colony formation, whereas overexpressing it and microRNA-143-3p simultaneously was able to counteract such promoting impact (Figures 4(b) and 4(c)). Transwell also demonstrated that microRNA-143-4p led to a reduction of TBX3-triggered cancer cell migration and invasion (Figure 4(d)). Based on western blot, TBX3 overexpression alone declined E-cadherin expression while elevating Vimentin and N-cadherin expression, hinting that those epithelial cells acquired mesenchymal properties. Nevertheless, such properties were reversed by microRNA-143-3p mimic (Figure 4(e)). Altogether, microRNA-143-3p restrained bladder cancer cell functions and EMT through downregulating TBX3.

## 4. Discussion

Tumor invasion and metastasis are complex processes involving many genes and steps [27]. EMT is one of the important behaviors of tumor metastasis [28, 29]. EMT is a biological process that greatly increases the invasion and metastasis of malignant tumors [30]. EMT mainly occurs in epithelial cell cancers, and therefore, it also regulates bladder cancer. In this context, we explored a molecular biomarker that may help us further understand the metastasis and invasion of bladder cancer in this study.

There is a study that proved that TBX3 is differentially upregulated in bladder cancer [20]. TBX3 expresses in any type of tissue during embryonic development and functions as a transcriptional inhibitor [31]. TBX3 is also involved in various carcinogenic processes, such as proliferation, migration, and invasion [32–34]. Moreover, TBX3 is closely relevant to EMT [35]. TBX3 can facilitate preinvasive breast cancer cell progression via stimulating EMT and upregulating SLUG [35]. TBX3 expression level is upregulated in many cancers, but most references focus on breast cancer instead of bladder cancer [36–38]. Hence, TBX3 was chosen for research. EMT-related protein expression level and cell biological behaviors were detected here by western blot and cell functional experiments, and the results verified the promotion of TBX3 on bladder cancer cell migration, invasion, and EMT. This indicated a good agreement between the above experiments and references that TBX3 acts as a promoter and is relevant to EMT in bladder cancer.

The article "MicroRNA-143-3p/TBX3 Axis Represses Malignant Cell Behaviors in Bladder Cancer" was retracted in 2023. Reasons: signs of a paper mill; suspected computer-generated content; unreliable results or conclusions; lack of ethics approval or compliance.

To further determine how TBX3 modulates bladder cancer progression, we predicted its upstream microRNA and performed correlation analysis. At last, microRNA-143-3p that had binding sites and was negatively correlated with TBX3 was obtained. MicroRNA-143-3p affects the development of various cancers as a tumor suppressor [39]. MicroRNA-143-3p expression is remarkably low and inhibits cell proliferation in colon cancer [40]. In breast cancer, microRNA-143-3p is less expressed which restrains the proliferation of breast cancer and stimulates apoptosis [41]. Similar phenomenon has also been observed in bladder cancer. SNHG1 is capable of endogenously sponging microRNA-143-3p in the cytoplasm of bladder cancer cells to affect cell proliferation and motor ability [42]. Likewise, we proved that microRNA-143-3p was notably less expressed and inhibited TBX3 expression in bladder cancer through experiments. In addition, rescue assay further presented that microRNA-143-3p overexpression downregulated TBX3 expression to mediate cancer cell migration, invasion, and EMT. EMT allows cancer cells to be equipped with mesenchymal properties to escape from primary tumors [43]. E-cadherin mediates signal transduction compound, loss of which is a clinical indicator of bad prognosis and metastasis [27]. It was posited that microRNA-143-3p/TBX3 axis hampered EMT to hinder bladder cancer migration and invasion. Such molecular mechanism was verified for the first time.

On the above, the microRNA-143-3p/TBX3 axis is closely related to bladder cancer migration, invasion, and EMT as evidenced by bioinformatics, molecular, and cellular analyses. In the future, we plan to further confirm our findings by animals and clinical trials and expect to provide more solid and perfect theoretical supports for bladder cancer diagnosis and treatment.

## Figures and Tables

**Figure 1:** TBX3 is markedly high in bladder cancer. (a) qRT-PCR detected TBX3 mRNA expression. (b) Western blot detected TBX3 protein expression level. All experiments were carried out in triplicate, and the results were expressed as the mean ± SD. Statistical significance was set when ∗ denotes *p* < 0.05, ∗∗ denotes *p* < 0.01, and ∗∗∗ denotes *p* < 0.001.

The article "MicroRNA-143-3p/TBX3 Axis Represses Malignant Cell Behaviors in Bladder Cancer" was retracted in 2023. Reasons: signs of a paper mill; suspected computer-generated content; unreliable results or conclusions; lack of ethics approval or compliance.

**Figure 2:** TBX3 facilitates EMT and cell functions in bladder cancer. (a) TBX2 transfection efficiency in T24 cells and BIU-87 cells in si-NC, si-TBX3, oe-NC, and oe-TBX3 groups. (b) CCK-8 assay indicated that silenced TBX3 remarkably inhibited T24 cell viability, while overexpressed TBX3 facilitated BIU-87 cell viability. (c) Colony formation assay indicated that silenced TBX3 remarkably inhibited T24 cell proliferation, while overexpressed TBX3 facilitated BIU-87 cell proliferation. (d) Transwell assay suggested that declined TBX3 expression suppressed T24 cell migration and invasion, while overexpressed TBX3 increased BIU-87 cell migration and invasion (100x). (e) Western blot detected TBX3, Vimentin, N-cadherin, and E-cadherin protein expression in each transfection group. ∗ denotes *p* < 0.05, ∗∗ denotes *p* < 0.01, and ∗∗∗ denotes *p* < 0.001.

**Figure 3:** MicroRNA-143-3p reduces TBX3 expression. (a) Intersection of downregulated microRNAs in bladder cancer and microRNAs with binding sites with TBX3. edgeR software was used (∣logFC | <1.5, FDR < 0.05) for differential analysis. Seven microRNAs were obtained. (b) Correlation analysis between the 7 microRNAs and TBX3. (c) Binding sites between two genes. (d) MicroRNA-143-3p targeted binding TBX3. (e) qRT-PCR detected microRNA-143-3p expression level. (f) MicroRNA-143-3p overexpression suppressed TBX3 mRNA expression. (g) MicroRNA-143-3p overexpression declined TBX3 protein expression level. ∗ denotes *p* < 0.05, ∗∗ denotes *p* < 0.01, and ∗∗∗ denotes *p* < 0.001.

**Figure 4:** MicroRNA-143-3p represses EMT and cell functions in bladder cancer via inhibiting TBX3 expression. (a) qRT-PCR detected TBX3 mRNA expression in each group. (b) CCK-8 detected cancer cell viability in each transfection group. (c) Colony formation assay detected cancer cell proliferation. (d) Transwell assay detected cell migration and invasion (100x). (e) Western blot detected TBX3 and EMT-related protein expression level in cancer cells in each transfection group. ∗ denotes *p* < 0.05, ∗∗ denotes *p* < 0.01, and ∗∗∗ denotes *p* < 0.001.

**Table 1:** qRT-PCR primer list.

Target gene	Primer (5′-3′)
MicroRNA-143-3p	F: GGGGTGAGATGAAGCACTG
	R: CAGTGCGTGTCGTGGAGT
U6	F: TGCGGGTGCTCGCTTCGGC
	R: CCAGTGCAGGGTCCGAGGT
TBX3	F: TTCCACATTGTAAGAGCCAATG
	R: CTTTGAGGTTCGTTGTCCCTAC
*β*-Actin	F: CTGGAACGGTGAAGGTGACA
	R: AAGGGACTTCCTGTAACAATGCA

## Data Availability

The data used to support the findings of this study are included within the article.
